# Arrhythmias Occurring in Children during HEMS Intervention: A Retrospective Cohort Study

**DOI:** 10.1155/2023/2974648

**Published:** 2023-11-23

**Authors:** Piotr Konrad Leszczyński, Arkadiusz Wejnarski, Patryk Rzońca, Angelika Gajowniczek, Robert Gałązkowski, Kryspin Mitura, Daryna Sholokhova

**Affiliations:** ^1^Faculty of Medical Sciences and Health Sciences, University of Siedlce, Siedlce, Poland; ^2^Department of Human Anatomy, Faculty of Health Sciences, Medical University of Warsaw, Warsaw, Poland; ^3^Emergency Medical Service, Mińsk Mazowiecki, Poland

## Abstract

**Background:**

Arrhythmias in patients during medical transport remain a challenge for medical personnel. Helicopter emergency medical service (HEMS) crews, as the only medical rescue teams in Poland to conduct rescue flights, keep detailed documentation of monitoring vital functions over short time intervals during the flight.

**Aims:**

The aim of this study was to determine the characteristics of cardiac arrhythmia in pediatric patients (up to 12 years of age) transported by HEMS operatives, considering life-threatening rhythms and those that occur during out-of-hospital cardiac arrest (OHCA).

**Methods:**

The analysis of HEMS medical documentation covered 90345 missions carried out from 2011 to 2020. Among all activations, 820 cases of arrhythmias in pediatric patients up to 12 years of age were extracted.

**Results:**

Missions for males accounted for 60% of all activations (*n* = 492), while flights for females accounted for 40% (*n* = 328). A statistically significant relationship between the number of HEMS flights and the season was demonstrated (*p* = 0.015). During the study period, pediatric patients mostly experienced cardiac arrhythmias in the form of supraventricular tachycardia (sVT) (*n* = 504). Asystole (*n* = 178) and pulseless electrical activity (PEA) (*n* = 52) ranked second and third in terms of occurrence, respectively. A statistically significant relationship between the type of heart rhythm disorder and age was demonstrated (*p* < 0.05).

**Conclusions:**

Heart rhythm disorders most often affected children between 0 and 3 years of age. As the patient's age increased, the incidence of arrhythmias decreased. Among pediatric patients, supraventricular tachycardia proved to be the predominant arrhythmia during the study period.

## 1. Introduction

Heart rhythm disorders are increasingly being detected in newborns, children, and adolescents, as new and more accurate methods of diagnosing abnormalities in the electrical function of the heart in pediatric patients become available. Arrhythmias may be asymptomatic, but in some cases, they cause serious life- and health-threatening consequences [1]. However, diagnostic and therapeutic options are limited in prehospital conditions, including the emergency care system. During medical rescues, the implementation of rapid treatment and the mitigation of negative consequences resulting from cardiovascular malfunctions are major challenges for medical personnel [2].

Among emergency medical teams, utilizing helicopter emergency medical services (HEMS) is the fastest option for transporting a patient to a medical facility. A HEMS crew in Poland consists of at least one professional pilot, a paramedic or nurse, and a doctor. The main tasks carried out by HEMS include the performance of medical rescue activities at the scene of the event and air ambulance transport to and between medical facilities [3].

Additionally, only HEMS crews use the National Advisory Committee for Aeronautics (NACA) score, which is a 7-point assessment of the patient's general condition. There are studies confirming the score's usefulness in transport carried out by HEMS [4, 5]. Based on the score, the patient's condition can be classified as severe (NACA 4), very severe (NACA 5-6), or moderate (NACA 3), and a decision can be made on which patients require immediate medical operations. The HEMS crew assesses the patient's condition using the NACA score to see if the patient is eligible for helicopter transport and whether there are no absolute contraindications (NACA 6-OHCA and NACA 7-death). Properly carried out classification of the patient leads to appropriate preparation for the mission, during which the crew needs to deal with a patient in severe or even critical condition and thus reduce the possibility of unwanted situations occurring during air transport. During the intervention, medical staff tries to ensure the presence and active participation of the child's guardian in rescue activities.

Arrhythmias in pediatric patients are most often related to tachyarrhythmias and bradyarrhythmias [6]. Attention should be paid to the criteria of heart rate, in which children differ significantly from adults and depend on age. Symptoms that may suggest arrhythmias are often nonspecific ailments, such as difficulty in feeding and anxiety or palpitations, heaviness in the chest, and presyncope [7]. Typical primary arrhythmias are atrial fibrillation (AF), atrial tachycardia (AT), atrioventricular nodal reentry tachycardia (AVNRT), atrioventricular re-entrant tachycardia (AVRT), bundle branch block (BBB), multifocal atrial tachycardia (MAT), permanent junctional reciprocating tachycardia (PJRT), supraventricular tachycardia (SVT), ventricular tachycardia (VT), and Wolff–Parkinson–White (WPW) [8]. The most common arrhythmias in children include sinus tachycardia, supraventricular tachycardia, bradycardia, and atrial fibrillation [9]. Atrioventricular blocks occur less frequently. Cardiac arrest mechanisms (ventricular fibrillation (VF), pulseless ventricular tachycardia (pVT), pulseless electrical activity (PEA), and asystole) are secondary rhythms.

The assessment of a patient with suspected arrhythmias includes a thorough family history and history and physical examination, followed by diagnostic testing. A 12- and/or 15-lead electrocardiogram, echocardiogram, exercise test, and home or ambulatory cardiac monitoring should be performed [10]. Unfortunately, in prehospital conditions, the diagnostic possibilities are significantly limited.

The Independent Public Health Care Air Ambulance Institution was established in 2000. The change in the name of the entity to “Polish Medical Air Rescue (PMAR)” occurred in 2016 as a result of the order of the Minister of Health on 9 November regarding the change of the name of the PMAR, which also granted it a statute [11, 12]. The current location of bases in Poland is shown in Figure 1. PMAR is a medical entity that aims to reach a patient in an emergency more quickly and to transport the patient to a hospital with an appropriate level of care. The role of HEMS in Poland, both in the urban agglomeration and in the countryside, has been confirmed by research [13–18].

There are insufficient data in the literature to characterize cardiac arrhythmias in prehospital pediatric patients. Their identification could improve the classification of health risks depending on age and type of event. The main objective of the authors of this study was to determine the types of cardiac arrhythmias in pediatric patients up to 12 years of age who received assistance from HEMS.

### 1.1. Specific Goals

- Characterization of the HEMS mission to pediatric patients
- Determination of cardiac arrhythmias in children, including cases of sudden cardiac arrest
- Analysis of pharmacological treatment in HEMS conditions

## 2. Methods

This retrospective study was carried out based on data provided by HEMS in Warsaw (Księżycowa 5, 01-934 Warsaw), taking into account medical documentation from the period 2011-2020. A group of 820 patients up to 12 years of age with cardiac arrhythmias was selected for this study from the total number of patients and the total number of missions among 90345 flights (Figure 2). Data on HEMS scene flights were analyzed. Data on the place of the event and the date were also analyzed. The following data were extracted from the patient information: age, sex, type of heart rhythm disorder, and clinical condition of the patient. Only cases with complete documentation were included in the analysis. The HEMS medical records contain rubrics defining the heart rhythm, which allowed for the exact determination of the type of arrhythmia examined by the emergency physician. The age threshold was adopted based on the ERC 2021 guidelines, which adopt a threshold of 12 years in PALS proceedings.

### 2.1. HEMS Equipment and Organization in Poland

Eurocopter EC135 helicopters are equipped with a transport defibrillator with a 12-lead electrocardiogram (ECG), noninvasive blood pressure (NIBP) monitor, 2 IBP monitors, adult and child respiratory therapy equipment, including neonatal, oxygen saturation (SpO_2_), and end-tidal carbon dioxide (EtCO_2_) equipment and a transport incubator (at selected bases), and certification in standards of advanced resuscitation procedures (advanced life support (ALS) and pediatric advanced life support (PALS)). Professional preparation of the patient for a flight and detailed monitoring during the mission are crucial for patient safety. Already at the stage of accepting the application for a pediatric patient, the crew tries to obtain information about the age and weight of the injured person. During the briefing, the crew determines the appropriate range of standards for the patient's basic vital signs and initially estimates the doses and dilution of drugs or the type and size of the necessary equipment. Data are verified on site events, e.g., using a dedicated pediatric emergency tape (org. Broselow Pediatric Emergency Tape). At the first contact with a pediatric patient, the crew tries to conduct an initial assessment, e.g., based on the PAT triangle (Pediatric Assessment Triangle 2020 American Heart Association). HEMS in Poland bases its procedures on the guidelines of the European Resuscitation Council. Children are a group of patients who require special attention due to anatomical, physiological, procedural, and legal specificities. Examination and necessary therapeutic interventions should be performed in accordance with the current recommendations of the European Resuscitation Council (ERC) in the field of PALS.

Legal basis for disposing of air medical rescue teams (Regulation of the Minister of Health) of August 19, 2019, on framework procedures for handling emergency notifications and notifications about events by a medical dispatcher is as follows [17]:

1. A statement that the time of reaching the scene of an emergency medical team other than an air medical rescue team is longer than that of an HEMS
2. When the time of transport of a person in a state of emergency by air from the scene of the event to a hospital emergency department or trauma center is shorter than the time of transport by emergency medical teams other than HEMS and may bring benefits in the further treatment process
3. When, in the opinion of the dispatcher, it is necessary

The HEMS team's readiness time depends on the time of day and night. The teams' response times are closely monitored by the navigation system:

(a) Time ready to take off during the day:
  - Within 60 km from base: until 3 minutes
  - Within a radius of more than 60 km to 130 km from base: until 6 minutes
  - Within a radius of more than 130 km from base: until 15 minutes
(b) Time ready to take off at night:
  - Within a radius of 60 km from base: until 15 minutes;
  - Within a radius of more than 60 km from base: until 30 minutes.

#### 2.1.1. Statistical Analysis

Data obtained in the process of documentation analysis were subjected to statistical analysis, which was performed using the STATISTICA program version 13.2 (Tibco Software Inc., Palo Alto, CA, United States). In the description of quantitative data, the means (M) and standard deviations (SDs) were used, and in the case of qualitative data, numbers (N) and percentages (%) were used. The Kolmogorov‒Smirnov and Lilliefors tests were used to verify the normality of the distribution of quantitative variables. The chi-squared test was used to assess significant differences between the analyzed qualitative variables. A nonparametric Kruskal‒Wallis test was used to investigate differences between more than two groups. The results were considered statistically significant at *p* < 0.05.

## 3. Results

### 3.1. Event Characterization

This study considered 820 HEMS interventions among pediatric patients up to 12 years of age with cardiac arrhythmias. In the analyzed period, the largest number of flights for pediatric patients with heart rhythm disorders occurred in 2019 (*n* = 125), which constituted 15.2% of all calls. However, the lowest number of flights was recorded in 2011 (*n* = 38; 4.6% of the total number of cases). A thorough analysis of HEMS missions, broken down by year, is included in Figure 3. HEMS flights (Table 1) were sent more often to rural areas (*n* = 440) than to urban areas (*n* = 380). Day flights were dominant, with 743 flights (90.6%), while night flights involved only 77 cases (9.4%). A statistically significant difference has been demonstrated between the season and the location of the incident (*p*=0.015). The analysis indicates that in rural areas, HEMS crews intervened more frequently during the summer (43.0% vs 35.0%), whereas in urban areas, this occurred during the winter (20.0% vs 12.5%) (Table 1). The highest number of flights was recorded in the summer (*n* = 322), and the lowest was recorded in the winter (*n* = 131). The number of patients that qualified for transport accounted for 619 people (75.5%), while 201 (24.5%) of the patients did not qualify for transport or were handed over to ground crews.

### 3.2. Patient Profiles

Forty percent (*n* = 328) of the affected individuals in the analyzed period were females, while 60.0% (*n* = 492) of those affected were males. The vast majority of patients were infants and neonates (*n* = 276; 33.7%). A detailed analysis of patients broken down by sex and age is presented in Figure 4.

The most frequently diagnosed conditions based on the ICD-10 classification in the analyzed patient group were injuries (30.4%), cardiac arrests (17.6%), and respiratory disorders (10.9%). Detailed results are presented in Figure 5. The most frequently occurring clinical symptoms within the studied patient group were apnea (36.0%), cyanosis (24.3%), dyspnea (14.6%), and signs and symptoms of shock (12.3%).

### 3.3. Heart Rhythm Disorders

In the study period, pediatric patients most commonly experienced cardiac arrhythmias in the form of supraventricular tachycardia (sVT) (*n* = 504). The least common heart rhythm disorder in children was atrioventricular (AV) block (*n* = 11). A detailed analysis of cardiac arrhythmias broken down by year is presented in Table 2.

The highest number of deaths occurred among pediatric patients under 1 year of age (*n* = 86 cases). However, the lowest number of deaths was recorded in the 4–6 age group (*n* = 16 cases). The conducted statistical analysis revealed a significant difference in mortality between infants under 1 year of age and children aged 1–3 years (31.2% vs 6.4%), as well as children aged 4–6 years (31.2% vs 15.5%).  Figure 6 presents a detailed analysis of the number of deaths with regard to a patient's age. Asystole was diagnosed most often in the age group below 1 year, which may be related to the mortality rate.

During the OHCA, asystole (*n* = 178) and pulseless electrical activity (PEA) (*n* = 52) ranked first and second in terms of number, respectively (Table 3). The conducted statistical analysis revealed significant differences in the NACA scale values depending on the presence of cardiac rhythm disturbances (*p* < 0.05). Higher NACA scale values were obtained in the case of bradycardia compared to supraventricular tachycardia (5.2 vs 4.3), AV block (5.2 vs 4.0), and atrial fibrillation/flutter (5.2 vs 4.4), as well as in the case of ventricular tachycardia compared to AV block (4.8 vs. 4.0) (Figure 7).

### 3.4. Pharmacological Treatment

Among patients with rhythm disorders who did not develop cardiac arrest (*n* = 578), the most commonly used drugs were analgesics (*n* = 261; 45.16%): fentanyl (*n* = 106; 18.34%) and morphine (*n* = 98; 16.96%). The second most frequently used group of drugs was benzodiazepines: midazolam (*n* = 154; 26.64%) and diazepam (*n* = 79; 13.67%). Catecholamines were used a total of 164 times: adrenaline (*n* = 129), norepinephrine (*n* = 20), and dopaminum (*n* = 15). Hypotensive medications were used 110 times (ephedrine *n* = 110). Target drugs for arrhythmias were administered 109 times: adenosine (*n* = 4), atropine (*n* = 80), and amiodarone (*n* = 25).

### 3.5. Medical Emergency Procedures

Depending on the patient's condition, the HEMS teams implemented specific medical rescue activities. In 271 cases, patients were sedated. In 587 patients, airway suctioning was necessary, followed by endotracheal intubation in 351 of all patients, and mechanical ventilation in 284 cases. Muscle relaxation was used in 108 patients, chest compressions were used in 258 children, and defibrillation was used in 35 patients (Table 4).

## 4. Discussion

Cardiac arrhythmias may occur in both adults and children. The correct heart rate depends on a person's age. For example, in newborns, the heart rate should be in the range of 120–160/minute, while in children aged 2 to 10, the norm is 60–110/minute, and in children over 10 years of age and adults, the norm is considered to be 60–100/minute. The pulse depends on the state of stimulation of a person; during sleep, it is lower, while during wakefulness, it is the highest [19]. Bradycardia means a slow heart rate, that is, a heart rate below normal with regard to the normal value depending on age. The main symptoms of bradycardia are apathy, dizziness, fainting, and drowsiness. Treatment of a child with a diagnosis of bradycardia most often involves pharmacotherapy or implantation of a pacemaker [20]. Tachycardia, on the other hand, concerns an excessively rapid heart rate. The main symptoms of tachycardia are palpitations, dizziness, and rapid breathing. Treatment of tachycardia depends on the clinical condition of the child and the type of tachyarrhythmia.

The following five elements should be noted in the ERC-suggested pediatric cardiovascular screening regimen:

1. Heart rate
2. Blood pressure
3. Pulse amplitude
4. Peripheral perfusion (capillary refill, skin color and temperature, and peripheral pulse deficit)
5. Preload (jugular veins, liver, and lungs).

Heart rate is a very important part of evaluating a baby. Therefore, it should be monitored continuously and reliably. The measurement of saturation alone with a pulse oximeter may be insufficient; first, because pulse oximetry is a method whose measurement can be quite easily disturbed, and second, the measurement result, averaged over a period of several seconds, reacts with a relatively large inertia. Therefore, children should always be monitored with both ECG and SpO_2_. In young children, mainly neonates and infants, reflex bradycardia occurs in response to hypoxia. In such a situation, the first action to be taken is to quickly oxygenate the child. The increase in oxygen saturation usually restores normal heart function quickly and does not require medication. On the other hand, a delay in improving ventilation caused, for example, by the preparation and administration of drugs, may lead to cardiac arrest. It should be remembered that in children, HR < 60/min, without signs of circulation, is treated as SCA. When helping a child, if possible, it is necessary to obtain as much information as possible at the scene of the incident, which may be helpful in the further treatment process. A checklist can help you to collect all data efficiently and comprehensively. Sometimes arrhythmias in children are asymptomatic and are detected accidentally, e.g., during a check-up [21]. Risk factors for arrhythmia include conditions such as fever, dehydration, infections, and inflammation [22]. For the purposes of this study, an attempt was made to analyze cardiac arrhythmias in pediatric patients up to 12 years of age who were HEMS patients. An increase in the number of interventions in the studied category of patients over the years (2011 = 38 vs. 2019 = 125) was observed. This may be due to the decision to create more bases where HEMS crew duty is 24 hours a day, as well as to an increase in the overall number of calls over the years. The number of flights operated by HEMS depended on the season. Many more flights were made in the summer than in the winter (summer = 322 vs. winter = 131). This may be due to the difference in weather conditions, the lack of a safe landing site, and the earlier nightfall in winter.

The number of patients qualified for transport by HEMS crews accounted for 619 people (75.5%). However, 201 patients did not qualify for transport. This may be due to the lack of indications for urgent air transport or failure to meet requirements (e.g., a patient currently experiencing cardiac arrest or with low chances of survival of air transport). The most common arrhythmia in pediatric patients was supraventricular tachycardia (*n* = 504), while children with AV block were the least reported (*n* = 11). The obtained results are confirmed by the study by Sacchetti et al. and the description of Jan KR et al., where the causes of ER sVT most commonly include tissue hypoxia, hypovolemia, fever, metabolic stress, trauma, pain, anxiety, toxins, anemia, and less common causes include cardiac tamponade, tension pneumothorax, and thromboembolism [23, 24]. The presence of tachycardia is sometimes adaptive to changing conditions inside or outside the body and is not always a consequence of heart disease (i.e., it may be a result of shock with different etiologies). The obtained results show a significant difference in the frequency of adenosine use compared to atropine (*n* = 4 vs. n = 80). It should be assumed that bradycardia in children is interpreted by HEMS doctors as an arrhythmia that poses a greater threat than accelerated heart rate. Tachycardia may manifest with regular or irregular heartbeat. The occurrence of tachyarrhythmia leads to a deterioration of hemodynamic performance and hypoxia of organs and tissues. sVT in some patients may present only with palpitations, while in others, there may be severe symptoms of tachycardia requiring rapid and intensive treatment and hospitalization. sVT is usually characterized in the ECG by a sudden onset and equally rapid end, a constant R-R interval, and abnormal P waves. When interviewing the legal guardians or parents of a child, it is often impossible to detect the cause, except for a previously experienced episode of sVT [25].

The next arrhythmias in terms of frequency of occurrence were asystole (*n* = 178) and PEA (*n* = 52). In pediatric patients, cardiac arrest occurs much more frequently when presenting asystole or PEA than when presenting VF/pVT. This was confirmed by the results of the work by Nordseth et al., which was carried out over 2006–2013 in a pediatric hospital in Philadelphia [26]. The study group consisted of 74 pediatric patients diagnosed with cardiac arrest. The study showed that 38.0% of patients had cardiac arrest presenting PEA and 16.0% presented asystole. Rhythms appropriate for defibrillation were observed only in 24.0% of the total cases. Such a low percentage of rhythms for defibrillation during resuscitation may result from the fact that in most children, cardiac arrest occurs in the respiratory mechanism or due to generalized body failure. On the other hand, cardiac arrest resulting from circulatory failure in children without congenital heart defects or cardiovascular diseases is rare. The most frequent cardiac arrhythmias were observed in children less than 1 year of age (*n* = 164; 28.4% of total arrhythmias in children). The incidence of arrhythmias decreased with the age of the child.

Sholokhova et al.showed that 60.0% of traumatic events among children occur among males [27]. The authors point out the dependence shown in the description of the patient's profile. The study group consisted of exactly 60.0% of male pediatric patients. In turn, the most common reason for HEMS calls were injuries (*n* = 249; 30.4%). Therefore, more frequent arrhythmias in males could be related to injuries suffered by children. This aspect requires further research.

The highest number of deaths occurred among pediatric patients younger than 1 year of age (*n* = 86). Such a high percentage of deaths may result from poorly developed organs and systems. Risk factors for early death include respiratory distress and respiratory failure, as the respiratory process of newborns and infants occurs only through the nose. Therefore, even a runny nose or a child being placed in an incorrect position to sleep can lead to respiratory arrest [28, 29].

### 4.1. Limitations of This Study

The authors see the need to conduct further studies on a larger group of children. The medical documentation analyzed retrospectively came only from the air ambulance base in Poland. There are no known outcomes for hospitalized patients or results of studies that could indicate the causes of cardiac arrhythmias. The authors performed a cross-sectional analysis of pathological ECG records of various etiologies, including rhythms associated with sudden cardiac arrest. The characteristics of prehospital emergency procedures do not allow for the indication of the causes of arrhythmias each time. The years 2021 and 2022 were not included in the study due to the confounding factor caused by the COVID-19 pandemic [28, 30].The study does not include other medical procedures due to space limitations and the main topic of the study. The HEMS doctor's documentation is completed manually and then transcribed into a digital database. This may result in incomplete or illegible data in cards that are difficult for the administrator to read.

## 5. Conclusions

The number of diagnosed cardiac arrhythmias in pediatric patients (up to 12 years of age) shows an upward trend in the last 10 years. The highest risk of death was found among children less than 1 year of age. Among patients with sudden cardiac arrest, the dominant ECG record was asystole, which potentially determines a worse prognosis. Only 12 patients (5.0%) of SCA-related rhythms presented with ventricular disturbances that were an indication for external defibrillation. The authors confirmed that nonshockable rhythms are statistically significantly more frequent during SCA in children.

Taking into account arrhythmias that may potentially require intervention in prehospital conditions (ventricular tachycardia, atrial fibrillation/atrial flutter, and AV block), their number is not significant (*n* = 35). Supraventricular tachycardia and bradycardia disorders may be secondary to the primary cause in pediatric patients (e.g., hypoxia and hypovolemia).

## Figures and Tables

**Figure 1:** Location of HEMS bases in Poland.

**Figure 2:** Selection of the study group according to PRISMA flow diagram.

**Figure 3:** HEMS missions to pediatric patients with significant cardiac arrhythmias by year.

**Figure 4:** Division of patients according to age and sex.

**Figure 5:** Diagnosis eventually made by HEMS crews.

**Figure 6:** Number of deaths recorded in each age group.

**Figure 7:** Correlation of the NACA score with cardiac arrhythmias.

**Table 1:** Division of flights considering the time of year and the place of the event.

Season of the year	All *n* (%)	Place of the event		
		Urban	Rural	*P* value
Spring *n* (%)	197 (24.0)	91 (24.0)	106 (24.1)	**0.015**
Summer *n* (%)	322 (39.3)	133 (35.0)	189 (43.0)	
Autumn *n* (%)	170 (20.7)	80 (21.1)	90 (20.5)	
Winter *n* (%)	131 (16.0)	76 (20.0)	55 (12.5)	

Bold value indicates its statistical significance.

**Table 2:** Type of heart rhythm disorder broken down by the age of patient (excluding OHCA).

Heart rhythm disorder	All *n* (%)	Patient's age (*n*)				
		Under 1 year	1–3 years	4–6 years	7–9 years	10–12 years
Supraventricular tachycardia *n* (%)	504 (87.2)	130	185	61	64	64
Ventricular tachycardia *n* (%)	12 (2.1)	6	2	1	2	1
Bradycardia *n* (%)	39 (6.7)	12	10	12	4	1
AV block *n* (%)	11 (1.9)	7	3	1	0	0
Atrial fibrillation/atrial flutter *n* (%)	12 (2.1)	9	3	0	0	0

**Table 3:** Sudden cardiac arrest (SCA) rhythms.

Rhythm of sudden cardiac arrest	All *n* (%)	Patient's age				
		Under 1 year	1–3 years	4–6 years	7–9 years	10–12 years
Asystole *n* (%)	178 (73.6)	90 (32.6)	22 (9.4)	15 (14.6)	27 (26.2)	24 (23.3)
PEA *n* (%)	52 (21.5)	16 (5.8)	10 (4.3)	12 (11.7)	5 (4.9)	9 (8.7)
VF/pVT *n* (%)	12 (5.0)	6 (2.2)	0 (0.0)	1 (1.0)	1 (1.0)	4 (3.9)

**Table 4:** Medical emergency procedures implemented by age of patient.

Medical emergency procedures	Under 1 year	Patient's age				
		1–3 years	4–6 years	7–9 years	10–12 years	*P* value
Sedation *n* (%)	121 (51.5)	50 (18.1)	43 (41.8)	28 (27.2)	29 (28.2)	0.000
Muscle relaxation *n* (%)	51 (21.7)	13 (4.7)	17 (16.5)	15 (14.6)	12 (11.7)	0.000
Defibrillation *n* (%)	2 (0.9)	13 (4.7)	4 (3.9)	12 (11.7)	4 (3.9)	0.000
Airway suctioning *n* (%)	168 (71.5)	196 (71.0)	71 (68.9)	72 (69.9)	80 (77.7)	0.659
Mechanical ventilation *n* (%)	83 (35.3)	77 (27.9)	44 (42.7)	41 (39.8)	39 (37.9)	0.037
Tracheal intubation *n* (%)	96 (40.9)	95 (34.4)	54 (52.4)	56 (54.4)	50 (48.5)	0.001
Chest compressions *n* (%)	38 (16.2)	109 (39.5)	34 (33.0)	40 (38.8)	37 (35.9)	0.000

## Data Availability

The data used in this study are available from the corresponding author upon request.

## Abbreviations

AF: Atrial fibrillation
ALS: Advanced life support
AT: Atrial tachycardia
AVNRT: Atrioventricular nodal reentry tachycardia
AVRT: Atrioventricular re-entrant tachycardia
BBB: Bundle branch block
ECG: Electrocardiogram
EtCO_2_: End-tidal carbon dioxide
HEMS: Helicopter emergency medical service
MAT: Multifocal atrial tachycardia
NACA: National Advisory Committee for Aeronautics
NIBP: Noninvasive blood pressure
OHCA: Out-of-hospital cardiac arrest
PALS: Pediatric advanced life support
PAT: Pediatric assessment triangle
PEA: Pulseless electrical activity
PJRT: Permanent junctional reciprocating tachycardia
PMAR: Polish medical air rescue
SCA: Sudden cardiac arrest
SpO_2_: Oxygen saturation
sVT: Supraventricular tachycardia
VF: Ventricular fibrillation
VT: Ventricular tachycardia
WPW: Wolff–Parkinson–White.

## Additional Points

*What is New*? The work presents a significant database from the national registry of helicopter emergency medical services (HEMS). The study covered cases from a period of 9 years, taking into account individual arrhythmias in pediatric patients in prehospital conditions. In the literature, there are insufficient data presenting the characteristics of cardiac arrhythmias in children in the prehospital setting. Their juxtaposition can help classify health hazards according to age and type of event. The novelty of the study is the determination of the types of cardiac arrhythmias in pediatric patients up to 12 years of age, who were helped by HEMS. The epidemiology of cardiac arrest was also indicated, with the distinction of the primary mechanism of the heart rhythm.
